The article "Hydrodynamic Cavitation: A Novel Non-Thermal Liquid Food Processing Technology" was retracted in 2024. Reasons: unreliable results or conclusions; a conflict of interest; concerns about the peer review.

# Hydrodynamic Cavitation: A Novel Non-Thermal Liquid Food Processing Technology

**DOI:** 10.3389/fnut.2022.843808

**Published:** 2022-03-04

**Authors:** Xun Sun, Weibin You, Yue Wu, Yang Tao, Joon Yong Yoon, Xinyan Zhang, Xiaoxu Xuan

**Affiliations:** ^1^Key Laboratory of High Efficiency and Clean Mechanical Manufacture, Ministry of Education, School of Mechanical Engineering, Shandong University, Jinan, China; ^2^National Demonstration Center for Experimental Mechanical Engineering Education, Shandong University, Jinan, China; ^3^Department of Mechanical Engineering, Faculty of Engineering, The University of Hong Kong, Hong Kong, Hong Kong SAR, China; ^4^School of Chemistry, The University of Melbourne, Melbourne, VIC, Australia; ^5^College of Food Science and Technology, Nanjing Agricultural University, Nanjing, China; ^6^Department of Mechanical Engineering, BK21 FOUR ERICA-ACE Center, Hanyang University, Ansan, South Korea; ^7^National Engineering Laboratory for Reducing Emissions From Coal Combustion, School of Energy and Power Engineering, Shandong University, Jinan, China

**Keywords:** non-thermal liquid food processing, sonochemistry, hydrodynamic cavitation, physicochemical property, microbial inactivation

## Abstract

Hydrodynamic cavitation (HC), as a novel non-thermal processing technology, has recently shown unique effects on the properties of various liquid foods. The extreme conditions of pressure at ~500 bar, local hotspots with ~5,000 K, and oxidation created by HC can help obtain characteristic products with high quality and special taste. Moreover, compared with other emerging non-thermal approaches, the feature of the HC phenomenon and its generation mechanism helps determine that HC is more suitable for industrial-scale processing. This mini-review summarizes the current knowledge of the recent advances in HC-based liquid food processing. The principle of HC is briefly introduced. The effectiveness of HC on the various physical (e.g., particle size, viscosity, temperature, and stability), chemical (nutrition loss), and biological characteristics (microorganism inactivation) of various liquid foods are evaluated. Finally, several recommendations for future research on the HC technique are provided.

## Introduction

To meet the expectation of today's consumers for foods with great taste, convenience, extended shelf life, low calorie, and high essential nutrients, the development of novel food processing technologies has always been the research focus (1), which is also part of the uprising Industrial Revolution 4.0 (2–4). Recently, to overcome the shortcoming of the conventional heating process, numerous researchers are focusing on several merging non-thermal technologies (e.g., high hydrostatic pressure, pulsed electric field, ultrasound, and cold plasma) (5, 6). Among them, hydrodynamic cavitation (HC) has been widely considered a promising non-thermal food processing technique. Except for the miraculous effect, the inherent scalability and practicability of HC make it suitable for industrial-scale productions. Even though HC-based food processing has been investigated for over 10 years, the amount of the relative research is relatively limited, and the recent progress is still not clear, which leads to no industrial example yet. To this, the present narrative mini-review explores these studies relating to food processing by HC, describes the influences of HC on the physical, chemical, and biological characteristics, and provides potential future directions for practice and research.

The article "Hydrodynamic Cavitation: A Novel Non-Thermal Liquid Food Processing Technology" was retracted in 2024. Reasons: unreliable results or conclusions; a conflict of interest; concerns about the peer review.

## Principle of Hydrodynamic Cavitation

Hydrodynamic cavitation is a rapid phase-changing phenomenon. When the pressure drops below the local saturated vapor pressure, the nuclei existing in liquid start to grow, triggered by the pressure difference between the inside and the outside of the bubble. Once the bubble undergoes pressure recovery or reaches its maximum diameter, it collapses and releases huge energy into the surrounding medium (Figure 1A) (9, 10). As a result, the sonochemical effect is induced at room conditions, which can be characterized by intense mechanical (shock wave and microjet with high pressure at ~500 bar and shear stress), thermal (local hotspot with ~5,000 K), and chemical effects (hydrogen and hydroxyl radicals). In addition, several secondary effects, e.g., mechanical vibration, turbulence, dispersion, emulsification, and macroscopic heating, can be generated (11, 12). Up to now, HC has shown promising performance and industrialization potential in various processes: water treatment (13), sludge disintegration (7), emulsification (8), biomass pretreatment (14), and food processing (15). Moreover, the extradentary conditions created by HC make it suitable to be effectively synergized with other intensification means including ultrasound, chemicals, plasma, or photo or electrochemistry.

**Figure 1:** Life cycle of a cavitation bubble **(A)** (7, 8), conventional non-rotational hydrodynamic cavitation reactor (NRHCRs) **(B)**, and representative advanced rotational HCRs (ARHCRs) **(C)**.

The hydrodynamic cavitation reactor (HCR), which is utilized to intentionally generate the HC phenomenon, is the most essential part of the HC technology because its performance determines the effectiveness and cost. By operational principle, HCR can be categorized as non-rotational and rotational types. Non-rotational HCRs (NRHCRs), such as Venturi, orifice, and vortex diode (Figure 1B), commonly generate cavitation in the contraction part and its downstream side is caused by pressure drop. They are utilized in most research regarding HC due to their simple structure and their ease of use. More detailed information on them can be found in many reviews such as Korpe and Rao (16), Bhat and Gogate (17), and Wang et al. (18). Advanced rotational HCRs (ARHCRs) that appeared recently (Figure 1C), where cavitation is induced by a high-speed rotating rotor, have demonstrated more superior performance in many applications, especially in food processing (1, 15), compared with conventional devices. Several researchers have been devoted to demonstrating their mechanisms by experimental [flow visualization (19–29) and vibration (20, 21, 26, 27) and thermal characteristics (19, 23, 28)] and numerical methods (30, 31). Nevertheless, the research on this emerging type of device is relatively limited even though it has been commercialized nowadays. Even though few researchers studied the effect of geometrical factors of ARHCRs on the performance (32) and optimized them (33), it is still far from complete (34), because the design methodology of ARHCR and the related process is absent, which requires further in-depth research in the future (35).

The article "Hydrodynamic Cavitation: A Novel Non-Thermal Liquid Food Processing Technology" was retracted in 2024. Reasons: unreliable results or conclusions; a conflict of interest; concerns about the peer review.

## Effect of HC in Food Processing

So far, HC has been successfully utilized for processing various categories of foods, such as juice, milk, jam, yogurt, or even ice cream. Due to the induced extraordinary conditions, the physical, chemical, and biological characteristics of foods can be significantly improved by HC. To intuitively demonstrate those effects, Table 1 summarizes several representative studies published recently.

**Table 1:** Overview of recent literature on the food processing by hydrodynamic cavitation (HC) (TSS, total soluble solid; SI, sedimentation index; TA, titratable acidity; TPC, total phenolic content; VC, vitamin C; AA, antioxidant activity; DPH, degree of protein hydrolysis; PME, pectin methyl esterase; TPC, total plate count; Y&M, yeast and molds).

**Food category**	**Treatment method**	**Volume (L)**	**Physical**								**Chemical**						**Biological** **(log reduction)**	**Additional** **information**	**References**
			**pH**	**particle** **size**	**viscosity**	**density**	**TSS**	**SI**	**color**	**TA**	**TPC**	**VC**	**AA**	**DPH**	**PME**	**TPC**	**Y&M**		
Orange juice	Orifice (*P_*in*_* = 4 bar, *T* = 70°C, *t* = 4 min)	1.5	–	H (–)^a^	L (–)^a^	–	–	H (+)	H		L (+)	H (–)	L (+)		H (–)	1.22	1.62	• The effect of HC on nutrition and enzyme was much lower than that of pasteurization • The effect of temperature (40–70°C) and duration (2–8 min) was studied	(27)
Orange juice	Orifice (*P_*in*_* = 5 bar, *T* = 33°C, *t* =15 min)	5	L (+)		M (–)^a^		L (–)		L	L (–)		L (–)	L (–)		L (–)			• The effect of HC on POD and PME was much lower than that of pasteurization • The energy consumption of HC (3.97 J/mL) was significantly lower than that of ultrasound (486 J/mL) and high pressure pulsed electric field (2,773 J/mL for 300 μs) • The effect of inlet pressure (3–15 bar) and duration (5–25 min) was studied	(31)
Sugarcane juice	Orifice (*P_*in*_* = 3.5 bar, *T_*final*_* = 50°C, *t* = 40 min)	8	L (–)		M (–)		M (–)		H	L (+)						3.3		• The effect of orifice structure, inlet pressure (2.5–3.5 bar), and duration (10–40 min) was studied	(32)
tomato juice	Orifice (*P_*drop*_* = 3–0 bar, *T* = 45–59°C, *t* = 10 min)	1.5		M (–)	H (+)			H (+)			L (–)							• Lycopene and phenolic contents were not altered after HC treatment • The microbiological quality was improved • The effect of inlet pressure (4–10 psi) and duration (5–15 min) was studied	(26)
Milk (Peanut)	Venturi (*P_*in*_* = 10 bar, *T_*final*_* = 50.1°C, *t* = 10 min)	1	L (+)	H (–)	H (–)		–	H (+)	M	H (–)				H (+)		1.19	0.3	• The optical microscopy results indicate that the fat globule size was significantly reduced by HC at high pressures • The effect of inlet pressure (6–10 bar) was studied • The effectiveness of HC and ultrasound was compared	(30)
Milk (raw)	Venturi (*P_*in*_* = 10 psi, *T_*final*_* = 47.93°C, *t* = 15 min)	1	L (+)	M (–)	L (+)		L (+)		M	M (–)				H (+)		0.93	0.98	• The effect of inlet pressure (4–10 psi) and duration (5–15 min) was studied • HC showed 21% energy efficiency with higher cavitational yield than ultrasound • For most cases, no separation was observed during the storage due to the reduced size of fat globules (from 6.3 to 3–2.2 μm)	(28)

a *H, high impact (>40%); M, medium impact (20–40%); L, low impact (< 20%), +, positive impact, –, negative impact*.

The article "Hydrodynamic Cavitation: A Novel Non-Thermal Liquid Food Processing Technology" was retracted in 2024. Reasons: unreliable results or conclusions; a conflict of interest; concerns about the peer review.

## Effect on Physical Characteristics

Several physical characteristics of foods (e.g., particle size, viscosity, and temperature) can be affected by HC.

The reduction in particle size, which results from the mechanical effect of HC, improves the homogenization of juices by modifying the physical structure, which leads to a lower rate of sedimentation and separation of sediments from serum and the increased apparent viscosity. For example, Terán Hilares et al. (36) found that the volume-based mean diameter [D (3, 5)] of tomato juice was decreased from 291 to 248 μm after only 4-min of HC treatment (reactor: orifice, volume: 1.5 L, pressure drop: 3–0.3 bar, temperature: 45–59°C), with a considerable increase in apparent viscosity from 5.59 to 19.8 cP at a shear rate of 105.6 s^−1^. In addition, HC-treated juice shows high stability with sedimentation index (SI) over 98% during 14-day storage at 5°C. Similar results can be also found in the treatment of orange juice by Arya et al. (37). For milk, like ultrasound, HC can disrupt the milk fat globule membrane, reduce the size of milk fat globule (MFG), increase the specific surface area of MFGs, and consequently promote the absorption through the walls of the small intestine. Pegu and Arya (38) found that a 15-min HC treatment (reactor: orifice, volume: 1 L, inlet pressure: 10 psi, outlet temperature: 47.93°C) reduced the size of MFG from 6.3 to 2.22 μm, whereas the high-temperature short-time (HTST) pasteurization did not affect this. In addition, the optical microscopic results show that the MFG of the HC-treated sample is considerably small and evenly distributed, compared with that of HTST. Nevertheless, the HC-induced reduction in MFG size is less than high-intensity ultrasound (HIU) where it can be reduced to <1 mm. This can be attributed to the high local energy density and the timescale of rarefaction–compression periods of HIU (39). Similar to HC-treated juices, the HC-treated milk is also stable and presented no phase separation even after 12 days of storage (38, 40). In addition, the mechanical effect also decreases the total soluble solid (TSS) content of liquid foods (37, 38, 40–42).

Viscosity is an important property of food that provides stability to suspended particles in foods and contributes to the mouthfeel (43). HC can cause a notable decrease in viscosity of blueberry (44), protein concentrate (45), milk (38), juice (42), and ice cream (46), etc. For instance, Li et al. (45) reduced the viscosity of milk protein concentrate from 211.76 to 93.35 mPa·s by HC treatment (reactor: ARHCR, volume: 4 L, rotational speed: 3,000 rpm). The authors conjectured that this may be because HC destroys the structure of protein gel, which results in a decrease in the elastic modulus of the proteins. They also found the solubility and wettability of the powder obtained from drying the concentrate. The results of the response surface methodology (RSM) in the study by Chen and Martynenko (47) show the existence of a strong positive correlation (*p* < 0.001) between viscosity and particle size, which indicates that the decrease in viscosity might also be due to the decrease in particle size (43). In addition, the rheological changes by HC also make less pseudoplastic or shear-thinning behavior of liquids (40), which results in less loss of the kinetic energy during the production process.

Due to the macroscopic thermal effect of HC, the liquid temperature can be continuously raised during HC treatments with relatively high thermal efficiency (i.e., the ratio of heating output to energy input): 20–40% for NRHCRs and 70–80% for ARHCRs (28). Such heating effect is particularly useful for food processing as it can synergize with HC to achieve a higher inactivation effect of microorganisms, without combining heating devices, which will be discussed later.

The article "Hydrodynamic Cavitation: A Novel Non-Thermal Liquid Food Processing Technology" was retracted in 2024. Reasons: unreliable results or conclusions; a conflict of interest; concerns about the peer review.

Except for the above effects, the influence of HC on the density, titratable acidity, and pH is negligible.

## Effect on Chemical Characteristics

To achieve better effectiveness, most HC-based works regarding food processing generally combine HC and heating treatments or directly use the heating effect generated from HC. Compared with traditional pasteurization, the negative effect of the HC or thermal process on the liquid foods is much lower, which indicates that more nutrients can be retained. Terán Hilares et al. (36) reported that, after the HC treatments with different outlet temperatures (35–62°C) and durations (0–10 min), no degradation of the lycopene content occurred in tomato juice at mild conditions. Moreover, the HC or thermal treatment can release chemicals with high thermal stability. Chen and Martynenko (47) found that the total phenolic contents, proanthocyanidins, and antioxidant activity of cranberry were maximumly increased by 40% (from 2.03 to 2.84 mg GAE/g), 32% (from 1.2 to 1.76 mg/g), and 48%, respectively, because they can be released from the fiber matrix and seeds and the partial depolymerization under HC and high-temperature conditions. Similar results can also be found in the studies by Chen and Martynenko (47) and Arya et al. (37).

Moreover, the HC or thermal treatment can also achieve a satisfactory removal effect on undesired thermostable enzymes, which are mainly associated with deterioration of juice quality. For instance, Arya et al. (37) achieved the 30–65% reduction of pectin methyl esterase (PME) in orange juice by HC (reactor: orifice, volume: 1.5 L, inlet pressure: 4 bar, duration: 4 min) under various treatment temperatures (40–70°C). In the study by Katariya et al. (41), the sole use of HC only reduced the peroxidase (POD) and PME from 3.19 to 2.75 Δ OD/mL and from 4.79 to 3.7 meq. H^+^ mL^−1^ min^−1^, respectively, which are far lower than that of pasteurization (reactor: orifice, volume: 5 L, inlet pressure: 5 bar, temperature: 33°C, duration: 15 min). For the blueberries containing polyphenol oxidase (PPO) and POD, Martynenko and Chen (48) completely inactivated the PPO and POD at 65°C and 80°C, respectively, without obvious loss of anthocyanins (reactor: Venturi, capacity: 5.5 kg). Moreover, the complete inactivation of enzymes results in the considerably long half-life of the HC-treated sample (i.e., 533.2 and 216.6 days for 4 and 20°C, respectively) than that of the pasteurized sample (i.e., 184.3 and 35 days for 4 and 25°C, respectively).

The article "Hydrodynamic Cavitation: A Novel Non-Thermal Liquid Food Processing Technology" was retracted in 2024. Reasons: unreliable results or conclusions; a conflict of interest; concerns about the peer review.

On the contrary, the nutrients can simultaneously suffer from both HC and thermal effects during the HC or thermal treatment, which leads to unfavorable nutrition losses, especially for thermosensitive contents. For example, as an antioxidant, vitamin C can react with hydroxyl radicals generated by HC. At the same time, vitamin C is also highly unstable during heat processing. Katariya et al. (41) utilize HC to treat orange juice at 5 bar for 15 min with a constant temperature at 33°C, and only a minor reduction in vitamin C (from 206 to 188 eq. μg AA/mL) was achieved. Nevertheless, when they combined HC with thermal treatment, the loss of vitamin C was significantly increased to 45.5, 61.1, 63.1, and 67.7% for 40°, 50°, 60°, and 70°C, respectively, with a fixed treatment time of 8 min, whereas these values are still lower than that of the pasteurization (69.5% at 90°C for 90 s) (37). As for proteins, the effect of HC or thermal treatment is relatively mild. Pegu and Arya (38) found that, after the HC treatment at an inlet pressure of 10 psi and an outlet temperature of 47.93°C for 15 min, the remained activity of alkaline phosphatase of HC-treated milk (1.17 μmol mL^−1^) is significantly higher than that of HTST-treated one (0.15 μmol mL^−1^). Sun et al. (49) found that the detrimental effect of HC or thermal treatment (70°C) on the nutritional composition of milk, i.e., mineral, fat, protein, and vitamin contents, is similar to that of the HTST method.

Regarding the effect on colors, because HC treatment can reduce MFG sizes and can result in a more homogeneous matrix and can consequently modify the light reflection, whiter color and higher lightness (L^*^ value) in milk can be generally achieved. In the study by Pegu and Arya (38), HC treatment increased the L^*^ value from 73.81 to 78.38, whereas the HTST reduced this value to 71.79 due to the partial whey protein denaturation and their aggregation to casein micelles. Salve et al. (40) found that the L^*^ value of HC-treated peanut milk (78.5–78.8) is slightly lower than that of untreated one (80.5), despite the fact that the average size of MFG was reduced from 0.27 to 0.16 μm (reactor: Venturi, volume: 1 L, inlet pressure: 6–10 bar, outlet temperature: 45.2–50.1°C, duration: 15 min). This may be because of the greater treatment time and temperature. For juices, the significant decrease and increase in the red-green value (i.e., a^*^, from 4.57 to 2.81) and L^*^ (from 30.6 to 32.8) of orange juice were demonstrated by Katariya et al. (41) at severe HC treatment with an inlet pressure of 13 bar. Except for the particle size reduction, the accelerated carotenoid isomerization of carotenoid pigment by HC can be a major reason for this. Arya et al. (37) observed that the HC-treated orange juice is more yellow and brighter, clear in appearance, which results from the rise in the yellowness (b^*^ value) from 34.66 to 41.75, whereas that of HTST-treated one is 29.08.

The article "Hydrodynamic Cavitation: A Novel Non-Thermal Liquid Food Processing Technology" was retracted in 2024. Reasons: unreliable results or conclusions; a conflict of interest; concerns about the peer review.

In summary, to achieve satisfactory treatment effectiveness, the intensity of HC and temperature has to be carefully compromised by comprehensively considering the nutrition loss and the benefit for each different case.

## Effect on Biological Characteristics

The improvement in the biological characteristics by HC is microbial inactivation, which is caused by the combination of mechanical, thermal, and chemical effects. The physical impact during the bubble collapse can lead to serious damage to cells (e.g., plasmolysis, membrane breakage, and cytoplasm) (50). In addition, because the microorganism travels with the high-speed flow, they can undergo collision when the flow impacts solid walls, which may result in cell cleavage (51). Thermal inactivation associated with membrane denaturation, ribosome aggregation, DNA strand breaks, and protein inactivation can be induced by hotspots (52). As for the chemical effect, various reactive oxygen species, generated from the radical chain reactions, can oxidize the sulfhydryl groups and double bonds in the proteins, lipids, and membrane surfaces (53). In the previous studies, HC maximumly achieved 3.3, 1.53, 1.42, 3.13, and 1.1 of log reductions in total plate count for sugarcane juice (42), peanut milk (40), orange juice (37), cranberry puree (47), and raw milk (39), respectively. More specifically, satisfactory inactivation effects on designated microorganisms can be obtained, such as alga [*Chlorella pyrenoidosa* (54), cyanobacterial (55), *Microcystis aeruginosa* (56), and *Pseudomonas aeruginosa* (57), etc.], bacteria [*Bacillus subtilis* (*B. subtilis*) (51), *Escherichia coli* (*E. coli*) (58), *Legionella pneumophila* (22), and *Staphylococcus aureus* (*S. aureus*) (58), etc.], yeast (59), and virus (60).

As mentioned in the above section, combining HC and thermal treatment can significantly increase the inactivation effect and reduce the required treatment duration. For example, Mane et al. (58) found that increasing the temperature from 28° to 50°C causes an increase in the disinfection rate of *S. aureus* by HC from 33.5% to 69.8%. Similar result can also be found in the study by Sun et al. (23), Sun et al. (53), Terán Hilares et al. (36), and Gregersen et al. (39).

The article "Hydrodynamic Cavitation: A Novel Non-Thermal Liquid Food Processing Technology" was retracted in 2024. Reasons: unreliable results or conclusions; a conflict of interest; concerns about the peer review.

Expect for the most widely utilized batch mode, HC with careful reactor design and optimal condition can gain satisfactory effectiveness in continuous mode, namely continuous HC (CHC). For instance, Sun et al. (49) utilized the CHC (ARHCR) to achieve 5.89, 5.53, and 2.99 ± 0.08 log reductions of *E. coli, S. aureus*, and *B. subtilis* inoculated in milk, respectively, at proper conditions. The subsequent safety evaluation indicates that the change in the concentrations of general bacteria and *E. coli*, and also the pH value and acidity of the CHC-treated milk stored at 5°C for 14 days is close to that of low-temperature long-time treated milk. Milly et al. (61–63) also obtained high log reductions (>6) for various pathogenic bacteria utilizing the CHC (ARHCR) without any support. The CHC not only greatly simplifies the whole production process but also reduces the processing time, resulting in lower loss of nutrition in foods. Nevertheless, such inactivation effect can only be achieved by ARHCRs, and conventional reactors are only suitable for batch mode.

More information on microbial inactivation by HC can be found in the reviews by Sun et al. (52) and Zupanc et al. (64).

## Conclusions and Future Perspectives

The present mini-review provides an overview of the novel HC technique for liquid food processing. The sonochemical effect of HC reduces the particle size and TSS, whereas the density, titratable acidity, and pH are less impacted. The negative effect of HC or thermal treatment at proper conditions on nutrition is much lower than traditional pasteurization. The complete inactivation of undesired enzymes can be achieved by HC, significantly increasing the shelf life. In addition, the HC-treated food demonstrates whiter colors, which may win the hearts and wallets of customers more easily. HC is highly destructive to various pathogenic bacteria. Therefore, HC can be considered a practicable technique for producing safe, healthy, and nutritious liquid foods with “fresh-picked” flavor with excellent physical stability.

Even though significant advance has been made to investigate HC food processing, it is still far from complete. Several challenges that should be seriously considered are outlined below.

(1) Most studies utilized commercial HCRs. Investigating HCR characteristics and establishing design criteria of HCR and its process by combining experimental and numerical methods are vital for the application of the HC technique. Moreover, the CHC is highly time-effective and flexible to integrate with existing conventional processes; thus, the development of ARHCR has to be intensely focused.
(2) The effect of HC on the physical, chemical, and biological characteristics is contradictory; therefore, optimizing several process parameters, such as cavitation intensity, duration, and temperature, is vital for producing high-quality foods. Moreover, because these parameters have a mutual influence on each other, it is important to reveal the interaction and synergism mechanisms in such a complex system. To arrange experiments in the most efficient way, Design of Experiments, e.g., RSM, has to be widely used.
(3) So far, most works have focused on applied research. Although the effectiveness of HC has been well-validated, the corresponding mechanisms are still needed to be further explored.

The article "Hydrodynamic Cavitation: A Novel Non-Thermal Liquid Food Processing Technology" was retracted in 2024. Reasons: unreliable results or conclusions; a conflict of interest; concerns about the peer review.

## Author Contributions

XS: investigation, writing original draft, and supervision. WY and XS: resources. YW, JY, XZ, XS, and XX: writing, reviewing, and editing. XZ and XS: conceptualization. All authors contributed to the article and approved the submitted version.

## Funding

This study was supported by the National Natural Science Foundation of China (Grant Nos. 51906125 and 52111540266), the China Postdoctoral Science Foundation (Grant Nos. 2020T130364 and 2019M650162), the Shandong Provincial Natural Science Foundation (Grant No. ZR2020KB004), the postdoctoral innovation project of Shandong Province (Grant Nos. 202002006 and 202101002), the Youth Interdisciplinary Science and Innovative Research Groups of Shandong University (Grant No. 2020QNQT014), the Hong Kong Scholars Program (Grant No. XJ2021030), and the National Research Foundation of Korea (Grant No. 2021K2A9A2A06039055).

## Conflict of Interest

The authors declare that the research was conducted in the absence of any commercial or financial relationships that could be construed as a potential conflict of interest.

## Publisher's Note

All claims expressed in this article are solely those of the authors and do not necessarily represent those of their affiliated organizations, or those of the publisher, the editors and the reviewers. Any product that may be evaluated in this article, or claim that may be made by its manufacturer, is not guaranteed or endorsed by the publisher.
